The article "Why Fish Oil Fails: A Comprehensive 21st Century Lipids-Based Physiologic Analysis" was retracted in 2014. Reason: a conflict of interest.

# Why Fish Oil Fails: A Comprehensive 21st Century Lipids-Based Physiologic Analysis

**DOI:** 10.1155/2014/495761

**Published:** 2014-01-16

**Authors:** B. S. Peskin

**Affiliations:** The International PEO Society, P.O. Box 56507, Houston, TX 77256, USA

## Abstract

The medical community suffered three significant fish oil failures/setbacks in 2013. Claims that fish oil's EPA/DHA would stop the progression of heart disease were crushed when The Risk and Prevention Study Collaborative Group (Italy) released a conclusive negative finding regarding fish oil for those patients with high risk factors but no previous myocardial infarction. Fish oil failed in all measures of CVD prevention—both primary and secondary. Another major 2013 setback occurred when fish oil's DHA was shown to significantly increase prostate cancer in men, in particular, high-grade prostate cancer, in the Selenium and Vitamin E Cancer Prevention Trial (SELECT) analysis by Brasky et al. Another monumental failure occurred in 2013 whereby fish oil's EPA/DHA failed to improve macular degeneration. In 2010, fish oil's EPA/DHA failed to help Alzheimer's victims, even those with low DHA levels. These are by no means isolated failures. The promise of fish oil and its so-called active ingredients EPA / DHA fails time and time again in clinical trials. This lipids-based physiologic review will explain precisely why there should have never been expectation for success. This review will focus on underpublicized lipid science with a focus on physiology.

## 1. Introduction

The object of this review is to show how there could be no possible expectation of general patient benefit with prophylactic fish oil use. It will be shown that the amount of EPA/DHA from routine fish oil recommendations is 20Xs–500Xs more than the body would naturally produce on its own from alpha-linolenic acid (ALA)—Parent omega-3.

Advances in quantitative analysis have been made in the 21st century which are not yet disseminated in the medical community; that is, the delta-6/-5 enzymes are not impaired in the general patient population, and the amount of EPA/DHA required on a daily basis by the brain is now known to be less than 7.2 mg/day. Neither extremely important fact was known in the 20th century.

Lipid physiology makes the following clear: (a) Marine oil's EPA/DHA spontaneously oxidizes at room temperature and more rapidly at normal body temperature—no level of antioxidants can stop this deleterious effect. (b) Fish oil blunts the insulin response and raises resting blood glucose levels. (c) Fish oil decreases critical prostacyclin (PGI2) in patients with atherosclerosis—a very bad outcome. (d) Fish oil rapidly decreases arterial compliance—increasing “hardening of the arteries.” (e) In contrast to researcher's expectations, fish oil accelerates metastases in animals. (g) Fish oil's EPA/DHA do nothing to increase cellular and tissue oxygenation; to the contrary, marine oils increase inflammation. (h) Marine oil consumption impairs mitochondrial functionality, making it an *anti*-antiaging substance.

The medical profession is unaware of or is not acknowledging the lipid science unequivocally showing the great harm that marine/fish oil's supraphysiologic amounts of EPA/DHA cause. As will be shown, the claim that prophylactic use of marine oil produces positive patient results is completely counter to 21st century lipid science.

## 2. Fish Oil Fails Extensively in Clinical Trials, but These Failures Are Often Underpublicized: Three Significant 2013 Fish Oil Failures

Since many medical professionals are under the wrong impression that fish oil incontrovertibly works, it is instructive to make clear there *are numerous recent and not so recent marine oil/fish oil failures occurring across all clinical areas.* There are more (underpublicized) failures than (supposed) successes. These failures should cause great pause.

Three highly significant fish oil failures occurred in 2013. In May 2013, The Risk and Prevention Study Collaborative Group (Italy) released a conclusive negative finding regarding fish oil for those patients with high risk factors but no previous myocardial infarction. Fish oil failed in all measures of cardiovascular disease (CVD) prevention—both primary and secondary [1]. This study was so conclusive that Eric Topol, MD, Editor-in-Chief of Medscape and Medscape's Heartwire for cardiologists, issued a new directive to patients to *stop taking fish oil*, that is, long-chain EFA metabolites of EPA/DHA [2]. The July 2013 landmark article published in the *Journal of the National Cancer Institute* entitled “Plasma Phospholipid Fatty Acids and Prostate Cancer Risk in the SELECT Trial” [3] confirmed prior post-2007 findings of increased prostate cancer risk among men with high blood concentrations of long-chain metabolites of *ω*-3 fatty acids from fish oil studies [4, 5]. The authors warned, “The consistency of these findings suggests that these fatty acids are involved in prostate tumorigenesis. Recommendations to increase *LC*ω*-3PUFA* (marine oil's EPA/DHA) intake should consider its *potential risks*.” The May 2013 trial [6] showed that macular degeneration victims were not helped by fish oil's significant DHA content. The year 2013 was very bad for fish oil findings. Why the failures?

## 3. Pre-2007 Studies Were Poorly Conducted and Inconsistent with the Science

In a 2012 meta-analysis regarding cardiovascular disease, reviewing 1,007 articles, only 14 studies met the criteria of randomization, double blindness, and placebo control [7]. Clearly, an enormous number of poorly conducted studies in the journals have conclusions that cannot be relied on and are misleading physicians and researchers worldwide. Studies should be used to confirm the physiologic, lipid science, not to be counter to it as many pre-2007 studies were.

In researchers' haste to offer patients a new, effective treatment, fish oil “successes” were highlighted and its failures downplayed. However, post-2007 “studies” of fish oil show significant accumulated failure [8]. When well-controlled studies and experiments are performed, as was done in Harvard Medical School's 1995 experiment giving one group of patients fish oil and a control group olive oil, CVD progression did not lessen with fish oil [9]. Fish oil fails; it has to as the science below confirms.

## 4. EFAs: Parent Essential Oils (PEOs) and Derivatives

There are only two true 18-chain carbon essential fatty acids (EFAs): linoleic acid (LA) with two double bonds and alpha-linolenic acid (ALA) with three double bonds. Neither can be manufactured in the body; both must come from food.

Longer-chain metabolites are synthesized from LA and ALA. These long-chain metabolites—not essential and often incorrectly termed “EFAs”—are correctly termed “derivatives.” For example, common derivatives of the omega-3 series are EPA (eicosapentaenoic acid) with five double bonds and DHA (docosahexaenoic acid) with six double bonds. To clarify the issue, I term LA and ALA “Parent Essential Oils” (PEOs) or “Parents.” I properly term all of their long-chain metabolites “derivatives.” The body makes these important derivatives from Parents “as needed” in *naturally minute amounts*. The literature often fails to clearly distinguish these two vastly different substances.

### 4.1. Most Parents Stay as Parents

A major mistake was made in the 20th century, which misdirected researchers. It was *wrongly assumed* that the vast majority of “Parents” would be converted into “derivatives.” This did not occur, causing the medical research community to proclaim that there were ubiquitous metabolic deficiencies impacting the delta-6 and delta-5 desaturase enzymes in the general population. This has been shown to be categorically false by advanced 21st century quantitative methods (described later). In humans, no more than one percent (1%) of Parents are *naturally converted* into derivatives. Fish oil mania wrongly (and hazardously) assumes the converse.

## 5. Fish Oil Impairs Normal Cellular Physiology: Pathophysiologic Disorders Are Expected

Theoretically (and in clinical experiments) fish oil supplements, in their “normal” although supraphysiologic amounts (calculated below), cause changes in membrane properties that impair oxygen transmission into and through the cell [10]. Physicians and other health professionals often prescribe these supraphysiologic amounts, deleteriously altering phospholipids of cell and mitochondrial membranes.

As will be detailed later, nonfunctional LA-based trans fats, oxidized LA entities, and* inappropriate omega-6/omega-3 ratios (caused in part from normally recommended, yet supraphysiologic, marine oil supplementation)* are all potential sources of unsaturated fatty acids—in particular, LA (Parent omega-6)—that can disrupt the normal membrane structure, significantly increasing the potential for cancer [11]. All of the supraphysiologic, excess EPA/DHA cannot be beta-oxidized away. Thus a significant amount of the excess will be physiologically incorporated into all cell membranes, detrimentally.

## 6. Arterial Intima: Endothelial Tissue Comprised of Epithelial Cells—CVD Explained

The innermost lining of arterial intima is endothelial tissue, comprised of epithelial cells containing significant LA, but no alpha-linolenic acid (ALA) [12, 13]. A significant biologic effect of oxidized LDL is its cytotoxic effect on cultured endothelial cells directly lining the arterial wall [14]. Dietary LA becomes adulterated (peroxidized) from food processing (described later) and deposited in arterial intimal cell membranes and leads to abnormal oxidation at the vascular injury site, thus causing injurious inflammation.

In this case, *abnormal oxidation,* caused by ex vivo radical induced lipid peroxidation (adulteration) of LA, involves formation of a hydroperoxide from LA by abstraction of a hydrogen atom as a radical from the doubly allylic methylene group between the two double bonds, followed by the addition of oxygen, a diradical, to make a hydroperoxide radical, which can then pick up another reactive hydrogen atom, perhaps from another LA molecule, to form the hydroperoxide. This, in turn, may break the O–O bond to form an alkoxide and a hydroxyl radical, which can continue to make more undesirable oxidized products [15]. Therefore, atherosclerosis can be prevented/arrested if endothelial cells remain fully functional [16].

Although lipid peroxidation can be caused by injury to tissue or aging, it does not have to be initiated in this fashion. Furthermore, a bivalent metal ion can cleave the O–O bond; nonfunctionality can occur from the commercial processing of the linoleic oil (LA).

## 7. Bis-Allylic Bonds: Fish Oil's Spontaneous Oxidation (Rancidity) at Room Temperature and In Vivo

Polyunsaturated fatty acids including LA contain the system HC=CH–CH_2_–CH=CH. Long-chain fatty acids contain *bis-allylic* hydrogens whereby the –C=C– units are separated by a single-bonded –C– (carbon) atom. The hydrogen atoms attached to each of these intermediate –C– atoms are called *bis-allylic* hydrogens and have the lowest C–H (weakest) bond-energies of the fatty acid chain. The weak bond makes them *enormously susceptible* to attack by reactive oxygen species (ROS) generated elsewhere in the body [17]. Because of the five double bonds in EPA and six double bonds in DPA, these metabolites are highly sensitive to temperature.

In particular, DHA, with its 6 double bonds, contains 5 bis-allylic bonds and is therefore *320 times more susceptible to oxidative attack*, that is, becoming rancid, than monounsaturated oleic acid (18 : 1), which has no bis-allylic hydrogens in its chain. A saturated fat membrane containing just 5% DHA (fish oil) is 16 times more susceptible to peroxidative damage [18]. Fish oil's DHA is 7 *times more susceptible* to peroxidative damage than LA (Parent omega-6), the most significant fatty acid by both weight and functionality in the cell's bilipid membrane. *The shifting of the body's antioxidants required to combat this physiologic insult causes a shortage elsewhere.* This fact should cause the medical community great concern. Keeping tissue fluid in frigid waters is not a physiologic concern of humans.

### 7.1. Marine Oils Keep Membranes of Fish Fluid in Frigid Waters

The following underpublicized medical fact goes a long way toward explaining marine oil's tremendous cancer- causing potential in humans. Fatty, cold-water fish (the type we are told is best) live in temperatures as low as 32°F, *but warm-water fish may live in 70*°*F waters and have 14Xs less EPA/DHA content than their cold-water relatives* [19]. At normal human physiologic temperatures, fish oil spontaneously becomes rancid (as the above section detailed).

A human placed in ice-cold, frigid waters would suffer hypothermia, freeze, and likely die. Fish do not freeze because they have significantly higher levels of the EFA derivatives EPA and DHA than those in humans.

Our ambient and physiologic conditions are not similar to that of fish. Marine/fish oil researchers did not consider this important fact. EPA/DHA acts as “biological antifreeze” to fish living in frigid waters. Humans do not require such copious amounts because we have an internal temperature of 98.6°F. The deleterious effects when humans consume supraphysiologic amounts of marine oil's EPA/DHA are described next.

## 8. Primary and Secondary Lipid Oxidation and Hydroperoxides

There is much to know regarding specific lipid oxidation markers. Oxidative rancidity occurs in 3 distinct stages/phases: initiation, propagation, and ultimately termination. During the initiation stage, molecular oxygen combines with unsaturated fatty acids to produce hydroperoxides and free radicals, both of which are very reactive. Heat and light increase the rate of all phases. Then, the products of this stage react with additional lipids to form other reactive chemical species—often termed “autooxidation.” In the final termination (secondary) phase, relatively unreactive compounds are formed, including hydrocarbons, aldehydes, and ketones. Quantitative measure of all phases is required for a complete picture.

### 8.1. Malondialdehyde (MDA)/p-Anisidine Increases with Fish Oil/Marine Oil

Supplementation with polyunsaturated fatty acids in particular, EPA/DHA, as opposed to saturated fatty acids, results in a *statistically significant increase in lipid peroxidation in the plasma and liver*. Fish oil ingestion raises levels of extremely harmful malondialdehyde (MDA) [20]: “Ingestion of CLO [cod liver oil] was associated with an increase in MDA excretion in all six subjects. The mean increase of 37.5%, from 24.5 ± 3.5 *μ*g to 34.7 ± 2.5 *μ*g MDA (mean + SEM), was [statistically] significant and CLO ingestion again was associated with *an increase in MDA excretion in all subjects.* The mean increase of 54.3%, from 31.7 *μ*g to 49.1 *μ*g MDA/sample was highly significant.” Parent omega-6 (LA) undergoes—like all PUFAs—lipid peroxidation, but the amount of MDA produced is much, much lower than that by oxidation of EPA or DHA because MDA production requires at least 3 or more double bonds in a molecule.

The p-anisidine test measures the aldehyde content generated during decomposition of hydroperoxides. It correlates well with volatile substances. Volatile aldehydes and other later-stage aldehydes leave behind a nonvolatile product that the p-anisidine test measures well (via correlation). “Pristine” *fish oil can have an allowable p-anisidine value of 19, clearly showing significant secondary stage oxidation* [21], whereas a PEO formulation *without fish oil is closer to a p-anisidine value of 4*—confirming fish oil's substantial inherent propensity to become rancid at room temperature.

### 8.2. Thiobarbituric Acid Reactive Substances (TBARS) Increase with Fish Oil/Marine Oil

A 2000 study reported in the *American Journal of Clinical Nutrition *found that plasma TBARS (substances which react to the organic compound thiobarbituric acid and which are a result of lipid peroxidation) were >*21% higher after fish-oil supplementation* than after sunflower-oil supplementation (containing Parent LA, not derivatives) and 23% higher than after safflower-oil supplementation (containing Parent LA, not derivatives). The article explored the limitations of the various assays available for the measurement of lipid peroxidation in vivo, including the F2-isoprostane assay's inability to provide direct information about the peroxidation of 20:5n-3 (EPA) and 22:6n-3 (DHA) [22]. Fish oil oxidizes in plasma, producing numerous deleterious products. This long-term damaging effect is cumulative.

### 8.3. Clinical Proof and Verification of Fish Oil's Harmful Oxidation

Regardless of antioxidant level added to the fish oil supplement, rancidity/peroxidation upon ingestion (in vivo) becomes a very significant and problematic issue. Oxidation of EPA leads to generation of a mixture of aldehydes, peroxides, and other oxidation products. Highly polyunsaturated, long-chained EPA and more so with DHA, due to its additional double bond, is readily oxidized at room temperature even in the absence of exogenous oxidizing reagents. Importantly, in vivo, a large increase in tissue and plasma accumulation of fatty acid oxidation products is noted in subjects consuming fish oil even after addition of antioxidant supplements to the diet—this effect strongly suggests extensive oxidation of omega-3 fatty acids such as EPA in vivo. This deleterious effect is true as evidenced by the trial in which a 14% decrease in life expectancy occurred in those animals fed fish oil [23].

In humans and primates such as the monkey, no quantity of in vivo antioxidants will stop EPA/DHA damage as measured by *lipofuscin*, the peroxidized “age spots.” Lipofuscin was three-fold (3Xs) greater in the livers of monkeys fed fish oil. Furthermore, another measure of oxidative damage, the levels of basal thiobarbituric acid reactive substances (TBARS), was four-fold (4Xs) greater than that of the monkeys fed corn oil with no EPA/DHA. The researchers found that even a ten-fold (10Xs) increase in alpha-tocopherol, a potent antioxidant, was not fully able to prevent the peroxidative damage from fish oil [24].

## 9. Inflammation and the Cancer Connection

As per the above details, oxidation of marine oil's EPA/DHA is inherently inflammatory. Inflammation is now seen as causal to cancer as it is to CVD: “The connection between inflammation and cancer has moved to center stage in the research arena” [25]. This rewriting of the textbooks comes from one of the world's most renowned cancer researchers, Robert Weinberg of MIT (originator of the term “oncogene”), causing him to revise his leading textbook, *The Biology of Cancer* (Garland Science, 2006), to reflect this new understanding.

Prior sections detailed how fish oil causes inflammation in vivo because EPA/DHA spontaneously oxidize at room temperature and much more quickly at body temperature. Their harmful hydroperoxide products become incorporated in esterified cholesterol and it is well known in cardiology that *oxidized* cholesterol causes the inflammation leading to CVD. Increased cancer is expected with increased consumption of marine oils.

The inflammation/cancer connection is supported with the finding that asbestos causes inflammation, reported in 2010 in *Medical News Today*. “For the past 40 years researchers have tried to understand why asbestos causes cancer. This research *emphasizes the role of inflammation* in causing different types of cancer” [26, 27].

Inflammation alone, regardless of initiating conditions, accelerates cancer proliferation. Since 2007, cancer researchers understand and acknowledge that the fundamental, *prime cause of cancer is inflammation*, not genetics [28–30]. A further inflammation/cancer connection was reported in *Cancer Epidemiology, Biomarkers & Prevention in 2005*, with the statement that “There is a growing body of evidence supporting the role of *chronic inflammation* with prostate carcinogenesis and thus the associations of transfatty acids with increased inflammatory response may explain their associations with prostate cancer risk” [31]. The SELECT [3] showed that marine oil's DHA was more inflammatory than trans fats.

## 10. Parent-to-Derivative Amounts and Metabolism

What percentage of PEOs does become converted (naturally) to long-chain metabolites such as EPA and DHA? This important question must be addressed and answered before their correct supplemental dosage (if any) can be determined. This fundamental research was neglected concerning marine oils, which tragically led to recommendations of *haphazard supraphysiologic overdoses* of marine oil's EPA/DHA.

New, twenty-first century quantitative research from both NIH and USDA shows considerably lesser amounts of natural DHA conversion/usage from ALA than the medical community has been led to believe. These findings will be upsetting to those health professionals recommending fish oil prophylactically. The conversion amount is much less than the medical field assumes: it is less than 5%—often less than 1%—with at least 95% of PEOs staying in Parent form. This singular mistake of assuming very high conversion amounts, whereas in actuality their conversion amounts are extremely low, led to the irrational fish oil mania.

Contrary to wrong dogma, the enzymes that produce PEO derivatives (the delta-6 and delta-5 desaturase enzymes) are *not impaired* in the vast majority of patients [32]. Conversion of ALA (Parent omega-3) to DHA is unlikely to *ever normally exceed 1% in humans* [33].

Research at the United States Department of Agriculture's USDA Food Composition Laboratory (2001) reported *a natural net conversion rate of a mere 0.046% of ALA to DHA and 0.2% to* EPA—not the highly misleading 15% conversion rate that is often quoted [34]. This is a mistake of nearly 2 orders of magnitude (100-fold). In 2009 NIH researchers determined the amount of DHA utilized in human brain tissue to be a mere 3.8 mg ± 1.7 mg/day. Therefore, based on the variance, brain tissue in 95% of all subjects, allowing for variation in brain size, would consume no more than 0.4 mg–7.2 mg of DHA per day [32].

### 10.1. No Delta-6/-5 Desaturase Widespread Impairment in (Average) Patients

Highly accurate, quantitative experiments were performed showing that both animals and the average healthy person are quite capable of metabolizing adequate amounts of DHA from Parent omega-3 (ALA).

As will be clearly demonstrated, there is no widespread impairment in the typical patient whatsoever; the normal conversion amounts are simply very low. *These conversion amounts are extremely small and naturally limited*. This mistake often leads to suprapharmacologic recommendations and can potentially overdose patients by factors of 20-fold to 500-fold, depending on specific supplement and amounts prescribed.

Because the body cannot oxidize away these tremendous overdoses of EPA/DHA, they become incorporated into tissue and organs with deleterious effects as confirmed by the skyrocketing increase in all epithelial-based cancers (described later). Supraphysiologic amounts are forced into tissue, causing gross physiologic imbalance and great potential for harm.

An important experiment measuring plasma fatty acids in 62 fire fighters concluded that the consumption of ALA-enriched (Parent omega-3) supplements over a 12-week period elevated levels of long-chain metabolites EPA and DHA. This experiment unequivocally showed the *unimpaired* effectiveness of ALA *conversion* from Parent omega-3. The researchers further stated that the general population could achieve the amounts of ALA required to obtain these effects by modifying their diet, ensuring adequate ALA (Parent omega-3) [35].

### 10.2. Vegans—Consuming No Fish—Produce Sufficient DHA

Even vegetarians consuming little or no fish had acceptable EPA/DHA levels [36]. This is a group that absolutely would be expected to manifest gross neurological abnormalities, including both visual impairment and cognitive impairment, yet there is no clinical evidence of such neurologic and cognitive abnormalities in vegetarians [36, 37].

Confirmation in 2010 showed that vegetarians with an intake of 0.3% DHA compared to fish eaters produced 85% of the EPA levels and 83% of the DHA levels that consumers of fish did. These amounts are within the “normal” ranges [37].

### 10.3. Rodents Have a 50-Fold Safety Margin: Would Not Humans?

Rats fed a DHA-free but *α*-LNA (n-3 PUFA) (Parent omega-3) adequate diet naturally produced from Parent omega-3 (ALA) fifty times (50Xs) more DHA than their brains required [38]—an enormous “safety factor.” Certainly, nature would ensure humans the same margin of safety shown to a rodent. This result in an animal species clearly supports highly quantitative 21st century research from the National Institutes of Health (NIH) finding extremely low—yet adequate—natural conversion rates in humans [32].

## 11. Amounts of EPA/DHA in Fish Oil Supplements: Pharmacological Plasma Overdoses

Given the above analyses, how much EPA/DHA does the typical marine oil/fish oil supplement provide? An average 1,000 mg health-food-grade fish oil capsule contains approximately 180 mg EPA and 120 mg DHA. Pharmaceutical-grade versions contain higher doses. Furthermore EPA ⇔ DHA. This is not the case with PEOs. They are unidirectional. The American Heart Association states that those with documented CHD are advised to consume about 1 gm (1,000 mg) of EPA + DHA per day. Is this advice rational? No.

As an example, using the USDA food composition research formulas covered earlier, if patients consumed a supplement of 600 mg of Parent ALA, they would naturally convert it to EPA by no more than the (generous) factor of 0.25% = 1.5 mg EPA and 1.5 mg × 0.63 × 0.37 = 0.35 mg to DHA in patient plasma. Therefore, just one capsule provides the amounts shown in the analysis below, and many people are overdosing even more by taking 2 to 4 fish oil capsules each day, likely in part because the cardiology and heart recommendations are often “EPA + DHA ranging from 0.5 to 1.8 grams per day.” What overdose does this translate to?

### 11.1. Potential EPA/DHA Overdoses Are Frequent

*Potential Overdose*  equates to the following plasma overdoses: EPA = 180 mg/1.5 mg = 120* times overdose* and DHA = 120 mg/0.35 mg = 340* times overdose*. These facts should cause great pause and concern. (Technically, a bit more is required for additional metabolic pathways aside from direct tissue incorporation like prostaglandin production, but it is not a significant amount by weight on a daily basis.) The medical community and most physicians and other health professionals may unknowingly be overdosing patients prophylactically with supraphysiologic supplemental amounts of omega-3 derivatives.

## 12. The Significant Problem: Radical Induced Lipid Peroxidation—Food Processors Require Long Shelf Life

Radical induced lipid peroxidation (adulteration) of omega-6 fats—in particular, LA—is created by food processors' need for long oil life during frying and baking, especially because their use of saturated fats is avoided. Omega-3 fats are never used in cooking; they are far too reactive.

Abnormal peroxidation of the Parent omega-6 oil (LA), therefore, is the core of the EFA-based deficiency. It has nothing to do with marine oils and everything to do with the adulteration of the plant-based Parent essential oil, LA. For example, trans fats—to some extent—are found in all commercial restaurants, supermarkets' prepared food and frozen food sections, and even in fine-dining restaurants' frying oils. The substrate for trans fats is Parent omega-6 (LA). Just 0.5 grams of a 1% trans fat containing adulterated oil (a conservative amount) is very harmful to humans. Even with the FDA's 2014 ban on trans fats, the FDA allows <0.5 grams/serving to be labeled as zero (0). Yet, this apparently negligible amount contains enough trans fats to overpower each cell in the body by a factor of approximately 3,600 [39].

### 12.1. Cellular Oxygenation Maximized with Unadulterated LA—Parent Omega-6

Marine/fish oils do nothing to promote cellular oxygenation in the mitochondria—this is a key role exclusive to Parent omega-6 (LA) [10, 40]. Marine oils, due to their inherent inflammatory property in vivo, cause the opposite of the desired effect and are therefore deleterious.

### 12.2. Pathophysiology Effects from Damaged Cell Membranes Caused by Radical Induced Lipid Peroxidation

With functional LA deficiency there is an enormous increase in permeability of epithelial tissue and an increase in capillary fragility, further explaining the pathophysiology of CVD and how it may be prevented [41]. Oxidation of LDL-C causes significant depletion of LA (Parent omega-6) [14]. Because LDL cholesterol is the transport vehicle for PEO delivery into the cell (described below), LDL cholesterol will transport LA into cells, whether the LA is defective or not (such as oxidized or trans entities).

Of great importance is the fact that with ingestion of marine/fish oil (EPA/DHA) there was a corresponding decrease in tissue's LA, causing pathophysiologic deficiency [42].

## 13. Tissue Incorporation of Dietary Fats is Proportional to Consumption

The concentration in adipose tissue triacylglycerols is *roughly proportional* to dietary concentration and is now frequently used as a *measure of relative dietary intake*. It has been long known that the fatty acid composition of the diet can influence membrane fatty acid composition [43, 44].

Fortunately, tissue alteration caused by supraphysiologic amounts of marine oil consumption can be remedied. Once removed, it takes 18 weeks to fully rid patients of the negative effects of fish oil [45].

## 14. Failure of LDL Cholesterol to Prevent CVD

It is now well known that LDL-C level, in and of itself, is not predictive of a cardiovascular event. This should not be a surprise, as the body has no plasma LDL-C sensor. This is not a “genetic defect” or oversight since the body has numerous sensors, such as for plasma blood glucose levels in nondiabetics, ranging from 70 to 90 mg/dL. This extremely tight tolerance of plasma glucose levels is 1 part in 1,000—approximately 0.1%. Since there is no hormonal-limiting metabolic factor for LDL-C, it must be viewed as a “dependent” variable, determined as a function of many other biological factors—not independent of them—as previously thought.

Studies confirm this fact. A review of a cholesterol/CVD causal effect categorically failed: among 12 populations with similar cholesterol levels clustered around “normal” levels—5.70 to 6.20 mmol per liter (220 to 240 mg per dL), the blood pressure readings and the *serum cholesterol levels were not predictive of ischemic heart disease mortality* [14]. If there were a causal correlation, then a 10% reduction should have had significant positive effects; it did not. Nothing has changed today regarding LDL-C's dismal success rate in both predicting and lowering patient CVD.

## 15. Lipids Are Variable in Tissue Composition

The significant variable in tissue is its lipid structure. Although the genetics of a particular species precisely specify cellular structure, its lipid composition can vary significantly—in particular, when suprapharmacologic amounts of long-chain metabolites are consumed, such as the case with fish oil supplements. A pharmacologic overdose cannot completely be oxidized away for energy or otherwise. Consequently, much of “the overdose” is forced into tissue composition, causing an improper structure—often in maintaining a linear relationship as does plasma and liver and as do RBCs [44, 46, 47]. Cellular bilipid membrane structure and its LDL-C structure warrant intense investigation.

Each of the approximately 100 trillion cells in the human body consists of a bilipid membrane. Importantly, PEOs comprise 25–33% of their polyunsaturated lipids [48]. Additionally, every mitochondrion, typically a hundred to thousands per cell, contains them, too [49, 50]. PEOs can be considered the “brick and mortar” of every cell, tissue, and organ, including mitochondria. In contrast, aside from the brain, eyes, and nervous system, most tissue and organs contain few derivatives like EPA/DHA.

## 16. Variability in LDL-C

The structure of LDL-C is complex. Its cholesteryl ester is key (Figure 1). The structure of cholesterol itself never changes, merely its esterified moiety—the acyl side chain. That is a big difference that many in the medical community may not appreciate. This is a simple condensation reaction, removing the water, catalyzed by the enzyme ACAT (acyl CoA: cholesterol acyl transferase) between a fatty acid and cholesterol. “R” symbolizes the hydrocarbon portion of the fatty acid. For example, if oleic acid were esterified with cholesterol, then R would be –C_8_H_17_=CH–C_7_H_14_ with the double bond in cis configuration.

Lipoproteins transport cholesterol and its esterified PEOs to the tissues via apoprotein B-100 (ApoB100).

Although the molecule itself may become oxidized, including its highly significant protein component (on a weight basis), that likelihood is extremely low. What is primarily oxidized are the fatty acids esterified to LDL-C (Figure 1) comprising the majority of the lipoprotein's center. Parent omega-6 quantities of esterified LA are approximately 85% of its overall 50% fatty acid content [51].

### 16.1. Esterified Cholesterol

The cholesteryl part or cholesteryl moiety is tied to a structure that does change—particularly, its EFA-based variable “R” component (Figure 1). It is well understood that the PEO LA dominates the esterified portion of cholesterol. The majority of the cholesteryl ester component is LA (Parent omega-6) [52].

The cholesterol ester portion is highly significant compared to free cholesterol or phospholipids (Figure 2). Approximately 70% of the cholesterol in the lipoproteins of the plasma is in the form of cholesterol esters attached to apolipoprotein B [53]. Of dietary cholesterol absorbed, 80%–90% is esterified with long-chain fatty acids in the intestinal mucosa [54].

### 16.2. LDL-C Is Highly Resistant to Oxidation in the Bloodstream

The fact that cholesterol itself is extremely resistant to oxidization is highly underpublicized, whereas its main esterified component, Parent omega-6 (LA), is more easily oxidized, especially ex vivo by food processing. Dietary LA that has already become oxidized prior to ingestion ex vivo is ubiquitous through processing of foods or overheating, since heating in the presence of air enhances peroxidation of PUFA glycerol esters [55, 56]. This insight suggests that looking in a new direction other than merely lowering LDL-C for the prevention of heart disease is warranted.

## 17. Human Antioxidant Levels Are Naturally Low

Normal antioxidant levels are lower than would be presumed to be adequate and normal if analysis were not performed in healthy patient populations as a control. The results are startling. Experiments show that the sum molar ratio of all *antioxidants to PUFA is a mere 1 : 165 (0.61%),* with *one antioxidant molecule having to protect the large number of 165 PUFA molecules* [51].

The total number of fatty acids bound in the different lipid classes of an LDL particle with a molecular mass of 2.5 million is on average 2,700, of which about one-half (1/2) are polyunsaturated fatty acids (PUFAs), mainly linoleic acid (Parent omega-6), with small amounts of arachidonic acid and docosahexaenoic acid (DHA). Furthermore, only minimal physical and chemical changes related to oxidation are produced by even a prolonged storage of LDL with oxygen or by incubation with low concentrations of copper ions.

Clearly, the quantity of naturally occurring antioxidants is too small for oxidation in vivo to be a significant physiologic issue [14, 51]. The sole logical conclusion is that the PUFA, in particular, LA, is being consumed and is entering the body in an already oxidized state caused by ubiquitous food processing.

## 18. New Insight: LDL-C Transports an Ingested “Poison”

### 18.1. CVD Explained: Processed Food Is the Culprit

Heating produces toxic products such as cholesterol oxides. If they are consumed—not produced in the body—they cause deleterious effects. Professor Gerhard Spiteller, who is Chairholder of Biochemistry, Institute of Organic Chemistry at the University of Bayreuth, Germany, has investigated EFAs and their degradation products—specifically, the influence of these substances on the physiology of mammals. He, too, concluded that *consumption of oxidized PUFA-cholesterol esters is responsible for the initial damage to endothelial cells* and that cholesterol oxidation products are incorporated into LDL cholesterol in the liver [57].

Given that both the cholesterol molecule itself is highly resistant to oxidation and Parent omega-6 is relatively resistant, the only acceptable conclusion is that the majority of the oxidized cholesterol damage is from its esterified component, that is, adulterated (oxidized) LA, patients unknowingly consume.

LDL then carries these toxic compounds into the endothelial walls where they cause cell damage. *Injury is not caused by an increase in free cholesterol but by an increase in cholesterol esters* of processed LA [58]. In atherosclerotic patients, LDL cholesterol is altered ex vivo by oxidation, and this altered LDL is taken up in unlimited amounts by macrophages. Dead macrophages filled with cholesterol's damaged, functionally impaired esters are then deposited in arteries. LDL-C is effectively transmitting a poison, that is, nonfunctional, adulterated, and harmful LA. We can now explain why statins fail.

### 18.2. Statin's Failure Explained

From the pharmaceutical company's own admission, the number needed to treat (NNT) for statins is no better than 60 over a 5-year period. This means that 60 patients would need to be treated for 5 years to see 1 positive outcome—*a 98.3% (59/60) failure rate*. Researchers often say that the NNT is much higher (worse). For example, JUPITER had an NNT of 95, meaning a 99% failure rate [59].

By statin's lowering of LDL-C, its esterified PEO component is also lowered, both adulterated (good outcome) and fully functional (bad outcome). This is problematic and precisely explains why statins do not work. By focusing on the ex vivo LA that has already become oxidized prior to ingestion through processing of foods, cooking, or overheating, a solution can be found to mitigate this damage.

## 19. Investigating Oils with respect to Arterial Health: IOWA Screening Experiment

A seminal screening experiment was conducted in 2010 comparing the effectiveness of PEO in increasing arterial compliance (flexibility) against fish oil [60]. This is a broad-based population screening—the most realistic population to see effectiveness, if any.

Arterial compliance is the most accurate physiologic assessment of a subject's cardiovascular health. Photoplethysmography is utilized with computer analysis of the (volumetric) curve's second derivative obtaining an acceleration curve. This output is compared to the database consisting of prior population scans grouped by age. The highly statistically significant results and excellent NNTs of IOWA confirm the theoretical predictions of both the failure of fish oil to increase arterial compliance and the significant (predictable) success of PEOs to improve arterial compliance across all populations.

### 19.1. Marine Oils Decrease Arterial Compliance: A Bad Outcome

The most remarkable finding was that subjects taking fish oil prior to PEOs obtained the most improvement. This was anticipated since those subjects started at a greater vascular deficit caused by the fish oil consumption.

Compared to PEOs, fish oil users had an “11-year-older” cardiovascular system as measured by arterial compliance population scans—more than a decade's additional “hardening of the arteries” compared to their physical age.

Ceasing fish oil use allowed the arterial system to revert to “normal” [45]. Once the vascular system was back to “normal,” the expected improvement from PEOs, as shown by the other groups, was also achieved, which translated to an even greater decrease in biological age based on where they had started. Clearly, fish oil accelerates vascular aging [60]. Marine oils are an *anti*-antiaging substance.

## 20. PEOs in Plasma, Lipids, and Esterified Cholesterol

It is necessary to analyze the Parent and derivative content of plasma lipids (lipoproteins, triglycerides, and esterified cholesterol) to determine the specific “bad actor” in CVD and cancer—every country's number 1 and number 2 killers—and confirm LA's prime importance. LDL's esterified linoleic acid is the major source for lipid peroxidation products, yet linoleic acid is highly resistant in LDL against oxidation [61]. This is critically important to understand.

With all the focus on omega-3 series fatty acids, both Parent and derivative, it is significant to note that the *free Parent fatty acids (nonesterified) in human plasma*, although minute in quantity, are ordinarily composed of about 15% LA (linoleic acid, Parent omega-6) and just 1% ALA (alpha-linolenic acid, Parent omega-3) [61].

Derivatives such as EPA/DHA are naturally much less significant in quantity than LA. In sharp contrast to the high amounts of n-6 series PUFAs, n-3 series PUFAs account for only 1.8% of the fatty acids in triglycerides, 3.5% in the phospholipids, and only 1.7% (ALA is 0.5%) in cholesterol esters. This high preponderance of LA is pervasive throughout: the LA/ALA ratio in triglycerides is 23 : 1; n-3 PUFA makes up only 1-2% of fatty acids in plasma [62]. Even in the brain, LA/ALA uptake is 100 times greater in favor of that of LA [62]. In the brain, AA, an omega-6 long-chain metabolite, comprises a significant 10% of the brain's long-chain fatty acids. Of particular importance is that the triglyceride stores concentrate the important Parent omega-6 fatty acid.

### 20.1. Importance of Parent Omega-6 and Prostaglandin Metabolites

In human lipid physiology, Parent omega-6 and its long-chain metabolites dominate over Parent omega-3 and its long-chain metabolites. The majority of the plasma fatty acids are LA (Parent omega-6) as are the triglyceride stores (adipose tissue). The metabolites of LA—in particular, prostaglandins PGE1 and PGI2 (prostacyclin)—are significant vasodilators. PGE1 is also the body's most potent anti-inflammatory. If functional LA bioavailability is lowered, the potential for inflammation will rise, leading to atherosclerosis. Weiss, for example, has noted that PGE1 (produced from functional Parent omega-6) reduces the fibrin deposition associated with the pathogenesis of atherosclerosis [63]. Membrane fluidity increases when more functional (undamaged) polyunsaturated fatty acids—in particular, linoleic acid—are available to incorporate into the membrane lipid bilayer.

Because LDL cholesterol is the transport vehicle for PEO delivery into the cell, LDL cholesterol will transport any LA into cells—defective or not—such as oxidized or trans entities. Mitigating the damage caused by extensive ex vivo intake of already oxidized LA is possible by supplemental ingestion of fully functional, unadulterated, nonoxidized LA.

## 21. Physiologic Excess of Omega-3 Series Fatty Acids Is Harmful, Decreasing Critical Omega-6 Series: Increases in CVD, Diabetes, and Cancer Are Expected

It was understood decades ago that consumed physiologic excess of omega-3 series PUFA is detrimental. Burns and Spector showed that the capacity of endothelial cells—relevant to carcinomas—and macrophages to release prostaglandins is reduced when they accumulate n-3 polyunsaturated fatty acids [64]. This is important because prostaglandins produced from PUFAs—in particular, Parent omega-6 (LA)—reduce the adhesion of tumor cells to microvascular endothelium. Most importantly, *fish oil is known to decrease critical anti-inflammatory PGE1 output in proportion to the amount of EPA/DHA consumed* [65].

### 21.1. Marine Oils Raise Resting Blood Glucose Levels and Blunt the Insulin Response Causing Insulin Resistance

Diabetes has become the world's number 1 epidemic. China has recently surpassed the USA in percentages of diabetics. Spontaneous autooxidation of blood glucose is a significant cause of diabetic patients' elevated increased risk of CVD. China has recently surpassed the USA in percentages of diabetics, and their consumption of marine oils keeps rising [66]. The negative impact marine oils have on diabetes, both Type I and Type II, is staggering.

Spontaneous autooxidation of blood glucose is a significant cause of diabetic patients' elevated increased risk of CVD, and marine oils increase plasma glucose levels. Both fish oil supplements and even “oily fish” itself are highly problematic for diabetics. In 2011, researchers looked at the effects on Type II diabetic patients consuming more fish. Only from *nonfatty* fish, containing more Parent omega-6 and much *less EPA/DHA*, did the experiment show *significantly decreased blood sugar* (good outcome). Further, those who ate “fatty” fish saw a decreased insulin output of 21% (bad outcome) compared to those not eating “fatty” fish [67].

*“Fatty” fish (containing more EPA/DHA), not a supplement, caused the elevated blood glucose*. EPA/DHA fish oil supplements cause elevated blood glucose and blunt the insulin response in diabetics. This deleterious finding was known years ago [68, 69]. Since “fatty/oily” fish caused the same deleterious effects as those of the supplement, the only logical conclusion is that fish oil—in any form—is harmful to any diabetic. Diabetes is America's number 1 epidemic and both oily fish and fish oil supplements exacerbate the condition. Furthermore, marine oils negatively impact the cellular membrane causing elevated insulin resistance. Because marine oils are known to displace critical Parent omega-6 in the cell membrane, this harmful effect is predictable. This issue impacts all tissue as shown below. Furthermore, it is well known cancer cells utilize glucose as their prime metabolic substrate (fuel). Oily fish and marine oil supplements—by allowing much greater blood glucose levels—both exacerbate patients' existing cancer metabolism and metastatic potential [40]. This effect is the opposite of any treatment's desired outcome.

### 21.2. Potential Brain Developmental Issue: Fish Oil Displaces Critical Omega-6 Metabolites Harming Tissue Structure

Importantly, fish oil potentially damages the brains of both infants and adults because critical omega-6 series metabolites are displaced [46]. This is another reason why fish oil failed to help Alzheimer's victims in a monumentally disappointing 2010 study [70]. The medical journal's authors specifically warned against feeding fish oil to human infants. This experiment was performed in rodents, but the results are applicable to humans because EFA metabolism is similar and applicable to both mammals and rodents [47]. Systemic rises in fish oil's EPA are largely compensated by decreased Parent omega-6 [42].

### 21.3. Fish Oil Causes Decreased Prostacyclin Production, Increasing CVD

Prostaglandins (hormone-like substances with extremely short half-lives not entering the bloodstream) are capable of both limiting thrombosis and reversing thrombosis in atherosclerotic patients [71].

Prostaglandin PGE1 is the body's most powerful anti-inflammatory and vasodilator and prostacyclin (PGI2) is a vasodilator and prevents both platelet adhesion and aggregation. These are both omega-6 metabolites.

Fish oil increases *endothelial* platelet aggregation in heart patients [72]. In patients with atherosclerosis, prostacyclin (produced in endothelial tissue) biosynthesis fell by a mean of 42% during the fish-oil period (extremely bad outcome). Synthesis of the platelet agonist thromboxane A2 (produced in the platelets) declined by 58% (good outcome). This may first appear to be a reasonably successful intervention, but that analysis would be incorrect for the following reason: atherosclerotic patients require increased intimal PGI2 output, as vessel wall thrombogenicity, and not reduced platelet adhesion, is a much more significant factor for minimizing thrombosis [73]. Furthermore, template-bleeding times were significantly prolonged in all fish-oil-consuming patients (bad outcome).

## 22. Association of Increased Marine Oils and Multiple Pathophysiologic Diseases 

### 22.1. Skin Cancer Has Become Epidemic as Fish Oil Supplement Consumption Increases and Results in Epidemics of Pathophysiologic Incorporation of DHA into Epithelial Tissue

The following associative speculation about marine oil's deleterious effects in the development of epithelial-based skin cancers requires confirmation. However, the physiologic/biochemical metabolic pathways detailing this conclusion are strong. Fish oil produces a pathophysiology in epithelial tissue, potentially leading to skin cancer. Likewise, adenocarcinoma of the prostate develops from aberrant epithelial cells. Are these conditions related? Logic tells us they are. We know there are no Parent omega-3 or omega-3 derivatives like EPA/DHA naturally occurring in epithelial tissue [12, 13]; therefore, any incorporation is supraphysiologic. Epithelial tissue's long-chain fatty acid composition is exclusive to Parent omega-6 (LA).

### 22.2. Increased Carcinoma with Increased Marine Oil Consumption: A Causal Relationship

A very strong melanoma/fish oil consumption association warrants attention. Skin cancer rates and fish oil consumption are both increasing. This is a very troubling (worldwide) association that must be addressed. Based on established physiology, it is predictable that the countries consuming the most fish-oil supplementation will contract skin cancer and prostate cancer the most—and they do, as will be shown later in this section. There are three quantitative EFA physiologic facts that must be understood in determining the definitive cause-effect relationship with fish oil use and cancer contraction. (A) There is neither Parent omega-3 (ALA) nor omega-3 long-chain metabolites (EPA/DHA) in epithelial tissue [12, 13]. (B) Each of the body's 100 trillion cells is comprised of a lipid bilayer with very little EPA/DHA, but significant LA and ALA (25–33%)—excepting those in epithelial tissue which is exclusively comprised of Parent omega-6 only (LA) [48, 49, 74, 75]. The same is true for the mitochondrion, except containing less ALA. Again, there is a physiologically negligible amount of EPA/DHA [49, 50]. We know *excess EPA/DHA displaces the main fatty acid in the membrane, Parent omega-6 (LA)* [46]. Is the (forced) incorporation of the derivatives EPA/DHA—by consumed supraphysiologic amounts—into epithelial tissue a direct cause of the increased skin cancer and therefore all epithelial-related cancers? The logical answer is yes.

Dermatologists are at a loss to explain the increase in skin cancer regardless of recommendations to their patients that they have less exposure to the sun. Human physiology strongly suggests that fish oil is a significant culprit. A seminal study in Norway revealed that *fish oil significantly increased the risk of skin cancer*. This is highly underpublicized, but reported in the *International Journal of Cancer* in 1997. Meticulous study (confirmed by pathology and cancer registry) of over 50,000 Norwegian men and women showed approximately a 3-fold increase in melanoma in women using cod liver oil (considered a superb fish oil supplement). The study was particularly strong, based on its unbiased approach, high participation and response rate, the fact that dietary data was collected prior to the onset of cancer, and the fact that each participant had a complete followup regarding occurrences of cancer, death, and emigration. In fact, all physicians and medical professionals in Norway are required to report malignant diseases to the Cancer Registry, and 98% of these cases are confirmed with microscopic tissue analysis [76]. In Norway, where fishing is a principal industry, they did not want to see a negative finding and it was not publicized. This study shows fish oil causing or associated with an increase in cancer—not prevention of cancer.

### 22.3. Epithelial (Skin) Cancers

The countries with the greatest skin cancer contraction rates, after Australia, are Scandinavia, Canada, and the United States [66]. Why is this? Marine/fish oil sales have constantly increased over the past 15 years and it has become America's number 1 supplement, and the rest of the world quickly follows America's dietary recommendations. Are these correlations mere coincidence? No. Based on the above science, they are predictable. Given that people are in the sun less and use sunscreen more, there are few valid reasons why skin cancer rates should be increasing worldwide and, in particular, these countries.

In 2010, *Cancer Research* published a historic article linking fish oil and increased colon cancer risk, as well as increased colitis [77, 78]. The researchers had hypothesized that “feeding fish oil enriched with DHA to mice would decrease the cancer risk,” but they found the opposite to be true. Instead, they discovered that the mice *developed deadly, late-stage colon cancer* when given high doses of *fish oil*. They observed *increased inflammation* and that, as a result, it only took just four weeks for the tumors to develop. This was true for mice that received the highest doses of DHA as well as those receiving lower doses. The researchers stated, “Our findings support a *growing body of literature implicating harmful effects of high doses of fish oil consumption in relation to certain diseases*.”

The researchers were shocked because they had relied on prior “studies,” not lipid (medical) science, to anticipate the effects of fish oil. Of particular importance was that these researchers even found low doses of fish oil to be harmful. In 2009, another significant journal article uncovered more problems with fish oil use, ultimately forcing the researchers to clearly state, “*The particularly high pro-metastatic effect of dietary n-3 PUFA on S11 cells rules out the generalisation that dietary n-3 PUFA inhibit tumour growth and progression*” [79].

### 22.4. Fish Oil Destroys Critical Mitochondrial Physiologic Functionality

Oncologists understand that mitochondrial functionality is a prime factor in the prevention of cancer. Yet, fish oil negatively impacts mitochondrial functionality. A seminal experiment appearing in *Cancer Cell* in 2006 is critical to the understanding of how fish oil causes such alarming mitochondrial damage, emphasizing that the connection is between fish oil consumption and cancer [80]. This test was conducted on live animals, not in a petri dish. Rats were fed fish oil or beef tallow. The scientists then examined the activity of critical mitochondrial enzymes from their kidney cells. The fish-oil-fed animals suffered an incredible 85% enzyme loss, while the beef-tallow-fed animals suffered only a 45% enzyme loss.

*Fish oil caused a 40% net additional reduction in critical mitochondrial enzyme production; that is, cellular respiration in the mitochondria is highly diminished*. Why would this be expected with supraphysiologic amounts of marine oils? Cardiolipin structure is highly compromised, as described next.

### 22.5. A Key Finding: All Tumors Suffer (Often Irreversible) Respiratory Damage

In remarkable research sponsored by the National Cancer Institute and published in 2008 and 2009, researchers found major abnormalities in content or composition of a complex lipid called *cardiolipin* (CL), stating these abnormalities are “*found in all tumors, linking abnormal CL to irreversible respiratory injury*” [81]. Cardiolipin is a fat-based complex phospholipid found in all mitochondrial membranes, almost exclusively in the inner membrane, and is intimately involved in maintaining mitochondrial functionality and membrane integrity. It is used for ATP (energy) synthesis and consists roughly of 20% lipids [82]. Nobel Prize-winner Otto Warburg, MD, PhD, first discovered the mitochondrial impairment/cancer causation link [40, 83–85].

With dietary marine/fish oil supplementation and its EPA/DHA modification of membrane fatty acid composition, which accelerates unnatural lipid peroxidation, significant effects of oxidative damage to many and varied cellular macromolecules occur. For example, peroxidized cardiolipin in the mitochondrial membrane can inactivate cytochrome oxidase by mechanisms similar to those of hydrogen peroxide as well as mechanisms unique to organic hydroperoxides. Dr. Hulbert warns, “*Lipid peroxidation should not be perceived solely as ‘damage to lipids,' but should also be considered as a significant endogenous source of damage to other cellular macromolecules, such as proteins and DNA (including mutations)*” [18].

Furthermore, the noncharged structure of aldehydes allows their migration with relative ease through hydrophobic membranes and hydrophilic cytosolic media, thereby *extending the migration distance far from the production site*. On the basis of these features alone, *these carbonyl compounds can be more destructive than free radicals and may have far-reaching damaging effects on target sites both within and outside membranes.*

Dr. Hulbert makes the importance of mitochondrial functionality clear with his statement, “The insight that the exceptionally long-living species, Homo sapiens, potentially provides for understanding the mechanisms determining animal longevity, is that the *fatty acid composition of mitochondrial membranes* may be much more important than the composition of other cellular membranes” [17]. A pharmacologic overdose of ALA metabolites exacerbates a shorter lifespan by altering the lipid (mitochondrial) membranes [23].

*Mitochondrial cardiolipin* molecules are targets of oxygen free radical attack, due to their high content of fatty acids—normally containing negligible long-chain omega-3 metabolites like DHA—*unless pharmacologically overdosed* as with marine/fish oil. Mitochondrial mediated ROS generation affects the activity of complex I, as well as complexes III and IV, via *peroxidation of cardiolipin* following oxyradical attack to its fatty acid constituents [18].

Most importantly, there is neither Parent omega-3 nor its metabolites in cardiolipin. Its main substrate is Parent omega-6 [18]. Alteration of mitochondrial structure by fish oil was known in 1990 and published at that time in an article in the *Proceedings of the National Academy of Science*, as follows: “Phospholipase A2 activity and *mitochondrial damage* are enhanced when *mitochondrial membranes* are enriched with *n-3 fatty acids* [from marine/fish oil]” [86].

Any cancer therapy not taking into account mitochondria efficiency and physiologic structural integrity is deficient and will fail in the long term, as Nobel Prize-winner Otto Warburg, MD, PhD, clearly demonstrated [83–85]. Others have expanded on his seminal discovery with a focus on cellular oxygenation [10, 40]. As confirmation of this fact, it is well supported that hypoxia in the prostate tumor causes greater tumor aggressiveness [87].

## 23. Furan Fatty Acids: Are Furan Fatty Acids Cardioprotective and Responsible for Any Positive Effects of Fish Consumption? 

In addition to abundant n-3 long-chain fatty acids, marine oil/fish oil contains furan fatty acids. Furan fatty acids (F-acids) are heterocyclic lipid components with a furan moiety in the center of the molecule, the predominate acid being F6 (C_22_H_38_O_3_). They are a large group of fatty acids characterized by a furan ring, which carries at one *α*-position an unbranched fatty acid chain with 9, 11, or 13 carbon atoms and at the other *α*-position a short straight-chain alkyl group with 3 or 5 carbon atoms. In most cases, two *β*-positions of the furan ring are substituted by either one or two methyl residues or other group. However, F-acid without any substitutions in both *β*-positions of the furan ring has also been found (in certain seed oils). They are labeled F_1_ to F_8_ with F_3_ and F_4_ being isomers. Algae, plants, and other microorganisms which produce furan fatty acids. There are only small amounts of these and they are often quite difficult to separate from other long-chain fatty acids.

Both marine and land animals consume F-acids, thereby incorporating these fatty acids into their phospholipids and cholesterol esters. These particular fatty acids are radical scavenging and may contribute to possible beneficial properties of fish consumption [88].

Recently, it was shown that this class of fatty acids efficiently rescues brain cell death induced by oxidative stress [89]. While the protective effect was strong, it was limited to an effective range only within the cell membrane. Regardless, this is still a significant effect and furan fatty acids should help reduce the risk of Alzheimer's disease.

Although promising, furan acids' effectiveness has been confirmed only in limited human controlled studies [90]. The significant issue to address is whether their effectiveness is countered by the inherent ability of supraphysiologic amounts of marine oil to spontaneously oxidize—per radical induced oxidation—as discussed in prior sections. We think so. Furthermore, furan fatty acids do not negate fatty fish's deleterious effects of elevating blood glucose and blunting the insulin response [67–69]. That is why, overall, the effectiveness of fish/marine oil in the amounts typically recommended is harmful; in particular, by elevating blood glucose levels in cancer victims. However, if the amount of marine/fish oil consumption is reduced significantly to normal physiologic levels as detailed per this review, there may be a positive role for marine oil.

## 24. Discussion

As demonstrated in cultures that consume fish, its consumption is fine. However, there are many cultures with excellent health and longevity that do not consume fish—the Hunza in Pakistan, the Vicambamba high in the Andes in Ecuador, the Abhasia of the Caucasus Mountains, and—in the United States—fully vegetarian 7th Day Adventists. *This review speaks solely of marine oil/fish oil supplements and the concentrated pharmaceuticals of concentrated DHA or EPA like Lovaza and Vascepa*. The medical profession is unaware or is not acknowledging the lipid science that unequivocally shows the great harm that marine/fish oil's recommended yet supraphysiologic amounts of EPA/DHA cause. This review gives the medical community many underpublicized physiologic facts that must be known and understood as the healthcare community revisits the practice of prescribing prophylactic marine oil to patients.

Fish oil cannot work, based on human physiology and biochemistry. Humans do not live in frigid waters where an “anti-freeze” is required, that is, EPA/DHA. These so-called active components spontaneously oxidize (radical induced oxidation) at room temperature and are even more problematic at physiologic body temperatures, causing numerous deleterious aldehyde secondary/end products regardless of antioxidant levels.

It has been clearly shown that the general population does not suffer impairment of delta-6/-5 desaturation enzyme impairments, as previously thought in the 20th century.

Prostate and other cancers along with CVD are predicted to increase in patients consuming fish oil on purely theoretical grounds, utilizing known physiology and biochemistry—and they do—in particular, epithelial cancers and impaired arterial intima.

Fully functional, Parent omega-6, LA, has been shown to be critical to both cellular oxygenation and mitochondrial function. Not distinguishing an adulterated (processed) EFA against a fully functional unprocessed EFA—in particular, LA—is the prime cause of confusion leading to inconsistent clinical trials on cardiovascular disease and cancer. The criticality of distinguishing between the effects of adulterated versus unadulterated forms of LA is obvious. Failure to do so has led to the incorrect and misleading conclusion that dietary intake of LA increases CVD risk, when it is only the *adulterated* LA that does [91]. The Parent EFAs are key; food processing is the root cause of EFA-related issues. Fish-oil supplementation has nothing to do with solving this issue. Although furan fatty acids found in fish oil are strongly radical scavenging, their quantities are too limited to counter the deleterious effects of supplemental marine/fish oils.

## 25. Conclusion

Marine/fish oil, in the supraphysiologic, prophylactic amounts often consumed, is harmful, possibly even more harmful than trans fats [3]. If proper physiologic amounts were utilized (<20 mg EPA/DHA), perhaps their furan acid content would be a significant positive factor; the concern of rampant oxidation is alleviated. Otherwise, given today's high quantities of fish oil recommendation, we see that their furan acid component is rendered ineffective. The medical profession needs to thoroughly review highly quantitative 21st century lipid physiology and biochemistry and offer the appropriate patient warnings. It is sincerely hoped that future researchers will approach the fish oil controversy with a more comprehensive grasp of the lipid biochemistry and physiology involved. Science must take precedence over “studies” which are often open to (mis)interpretation, leading to continual reversals and inconsistent results in clinical trials.

Using the most direct and effective physiologic measure, fish oil in the doses suggested is unequivocally shown to be an *anti*-antiaging substance, *increasing vascular “biologic aging*” by over a decade—causing “hardening of the arteries”—compared to PEO consumption. *Compared to taking nothing, fish oil decreased subjects' arterial compliance (a bad outcome), by nearly four years* [60].

Prophylactic marine oil consumption given its supraphysiologic EPA/DHA amounts—both theoretically and in clinical use—leads to increased inflammation, increased CVD, and increased cancer risk.

## Figures and Tables

**Figure 1:** Cholesteryl ester.

**Figure 2:** Structure and composition of a low-density lipoprotein showing the significance of its esterified cholesterol structure in its center (with permission, *Textbook of Medical Physiology (9*th* edition)*, page 874, 1996, W. B. Saunders Company).
